# Radioactive Iodine Ablation Can Reduce the Structural Recurrence Rate of Intermediate-Risk Papillary Thyroid Microcarcinoma: A Meta-Analysis

**DOI:** 10.1155/2022/8028846

**Published:** 2022-09-06

**Authors:** Min Zhao, Xinyu Shi, Jing Zhang, Shengming Deng, Yeye Zhou, Runze Wen, Yixing Lu, Bin Zhang

**Affiliations:** ^1^Department of Nuclear Medicine, The First Affiliated Hospital of Soochow University, No. 188 Shizi Street, Suzhou 215006, China; ^2^Department of General Surgery, The First Affiliated Hospital of Soochow University, No. 188 Shizi Street, Suzhou 215006, China

## Abstract

**Background:**

The incidence of papillary thyroid microcarcinoma (PTMC) has significantly increased in recent years, and the decision to use radioactive iodine (RAI) ablation in low-risk (LR) and intermediate-risk (IR) patients is controversial. The aim of this study was to evaluate whether RAI ablation can reduce the recurrence rate in LR-IR PTMC patients.

**Methods:**

A comprehensive literature search of the PubMed, Embase, Cochrane Library, and Web of Science was conducted according to the PRISMA statement.

**Results:**

There were 8 studies in English that fit our search strategy, and a total of 2847 patients were evaluated. The results of the meta-analysis showed RAI ablation in LR-IR PTMC patients did not reduce cancer recurrence (risk radio (RR) 0.56, 95% CI 0.19-1.70, *P* = 0.31). Nevertheless, we further performed data analysis and found that IR PTMC patients without RAI ablation had a higher rate of cancer recurrence than those who underwent RAI ablation (RR 0.23, 95% CI 0.11-0.49, *P* = 0.0001). Furthermore, patients with risk factors for lymph node metastasis (RR 0.16, 95% CI 0.06-0.42, *P* = 0.0002), microscopic extrathyroidal extension (RR 0.19, 95% CI 0.06-0.60, *P* = 0.005), and multifocality (RR 0.13, 95% CI 0.04-0.45, *P* = 0.001) in the absence of RAI ablation were more likely to have recurrence.

**Conclusions:**

Based on our current evidence, RAI ablation can reduce the cancer recurrence rate over 5 years in IR PTMC patients, especially when patients have some risk factors, such as lymph node metastasis, microscopic extrathyroidal extension, and multifocality.

## 1. Introduction

According to the World Health Organization (WHO), the incidence of papillary thyroid microcarcinoma (PTMC) with dimensions of 10 mm or smaller has significantly increased in recent years [1, 2]. Although the majority of patients with PTMC have a good prognosis, disease recurrence after initial treatment does occur. Locoregional recurrence and even distant metastasis have been reported in some patients with PTMC treated with surgery [2–6].

The American Thyroid Association (ATA) risk of recurrence stratification approach is often used to classify each PTMC patients as low, intermediate, or high risk [7]. Intrathyroidal PTMC without signs of extrathyroidal extension, vascular invasion, or metastasis is regarded as low-risk. Microscopic extrathyroidal extension and lymph node metastasis are seen in intermediate-risk individuals. High-risk patients have macroscopic extrathyroidal extension, inadequate tumor excision, and distant metastasis.

Radioactive iodine (RAI) ablation after total or near-total thyroidectomy (TT/NT) is one of the current measures for the treatment of PTMC. The aim is to ablate any residual thyroid tissue and any small residual tumors to limit the possibility of cancer recurrence or metastasis [8]. The incidence of PTMC has increased rapidly in recent years, giving rise to controversy over treatment strategies. Some experts believe that the term “microscopic” does not indicate a low-risk malignancy. Therefore, they advocate extensive surgery, as well as postoperative RAI ablation, which can significantly decrease the recurrence rate of patients [9, 10]. In contrast, some specialists suggest that RAI ablation after surgery may be overtreatment for LR-IR PTMC patients [11, 12].

According to the 2015 ATA guidelines [7], RAI therapy is recommended for high-risk patients with macroscopic extrathyroidal extension, distant metastasis, or incomplete tumor resection. As for PTMC without adverse features, RAI ablation is not recommended. It remains unclear whether RAI ablation in LR-IR PTMC patients reduces recurrence. Thus, we used a meta-analysis to clarify the value of RAI ablation in cancer recurrence in LR-IR PTMC patients. We present the following article in accordance with the PRISMA reporting checklist.

## 2. Materials and Methods

The PRISMA (Preferred Reporting Items for Systematic Reviews and Meta-Analyses) guideline [13, 14] was used to perform the systematic review. We have followed the protocol that was registered in INPLASY (INPLASY202220030).

### 2.1. Search Strategy

We used the following search method to search the PubMed, Embase, and Cochrane library through December 2021: (“remnant ablation”[tiab] OR “radioiodine”[tiab] OR “radioactive iodine”[tiab] OR “iodine 131”[tiab] OR “iodine-131”[tiab] OR “RAI” [tiab]) AND (“papillary thyroid microcarcinoma” [tiab] OR “papillary microcarcinoma” [tiab] OR “thyroid microcarcinoma” [tiab] OR “PTMC”[tiab]). The most recent search took place in December 2021. Only studies that were published in English with a complete text were considered. When many publications reported findings from the same patients, the most recent or comprehensive study was selected.

### 2.2. Inclusion and Exclusion Criteria

Articles that met the requirements were identified based on the flow chart in Figure 1. The criteria for inclusion in the study were as follows: (1) LR and IR PTMC patients who are in a disease-free state after TT/NT, (2) with RAI ablation vs. without RAI ablation groups, and (3) reporting of the outcome of cancer recurrence. Studies were excluded if (1) high-risk patients with macroscopic extrathyroidal extension, distant metastasis, or incomplete tumor resection; (2) patients with biochemical recurrence; (3) with a median follow-up period of less than 5 years; and (4) lacking any necessary data.

### 2.3. Data Extraction

Two of the researchers independently assessed all the selected papers to see if the articles met the requirements. The two authors resolve any differences that arise through discussion. If no agreement is reached, the other authors are contacted, and a decision by popular election is taken.

The following information was extracted according to a fixed protocol: first author's name, publication year of the article, geographical location, demographic information (age and sex), pathological characteristics of PTMC, follow-up time, and endpoint. The endpoint was defined as the recurrence rate between with or without RAI ablation therapy after TT/NT, as defined by each eligible study. In this meta-analysis, recurrence is divided into locoregional recurrence and distant metastasis. Recurrence was defined as structural recurrence after completion of initial treatment and identified using imaging modalities, such as ultrasonography, diagnostic radioactive iodine scan, PET scan, or MRI scan, followed by cytological or histological confirmation, regardless of serum levels of thyroglobulin (Tg).

### 2.4. Statistical Analysis

The meta-analysis was performed using Review Manager (RevMan) version 5.4. Dichotomous data were compared using a relative ratio (RR), and 95% confidence intervals (CI) were calculated for each estimate. A *P* value of < 0.05 was considered statistically significant. We determined heterogeneity by visual inspection of forest plots and using the *χ*^2^ test and *I*^2^ statistic. More specifically, when *P* < 0.10 and *I*^2^ > 50%, there is statistical heterogeneity and a random-effects model should be used, otherwise, a fixed-effects model was chosen. When we found heterogeneity, we attempted to determine potential reasons for it by examining individual study and subgroup characteristics.

### 2.5. Quality Assessment

The Newcastle-Ottawa Scale (NOS) [15] was used by two reviewers to independently evaluate the quality of retrospective (case-control and cohort) researches. The NOS is made up of three components: patient selection, comparability of research groups, and assessment of exposure/outcome. A total of nine objects were retrieved, and each object was assigned a score of one. Overall, the ratings ranged from 0 to 9. If the ratings were more than or equivalent to 5, the paper was deemed of good quality. Any differences amongst authors were resolved by a reassessment of the initial paper as a whole.

## 3. Results

### 3.1. Study Selection and Characteristics

The abovementioned search strategy yielded no randomized controlled trials. As shown in Figure 1, out of 898 findings, 8 studies met the inclusion/exclusion criteria for this study [16–23].

In the eight included studies, there were 2874 PTMC patients with a median follow-up time ranging from 5.3 to 8.4 years. Of these patients, 1742 received RAI ablation at doses ranging from 30 to 150 mCi. The detailed characteristics of the included studies are given in Table 1.

### 3.2. The Methodological Quality of Included Studies

Table 2 shows the results of the quality evaluation according to the NOS. The comprehensive search tactics generated 8 retrospective studies, all of which were judged to be of high quality: three studies received a NOS score of 9 [17, 18, 21], and five studies received a NOS score of 8 [16, 19, 20, 22, 23].

### 3.3. Meta-Analysis Findings

#### 3.3.1. Cancer Recurrence Rate in the Overall Population

Cancer recurrence in patients treated with or without RAI ablation after TT/NT was compared. In the overall population, the cancer recurrence rate in patients treated with RAI ablation (2.87%) was lower than without RAI ablation (3.53%). The heterogeneity was found between different studies (*I*^2^ = 76%, *P* = 0.0004), and the random effect model was used (RR 0.56, CI 0.19-1.70, *P* = 0.31). Unfortunately, there was no statistically significant difference between these two groups (Figure 2). When cancer recurrence was divided into locoregional recurrence and distant metastasis, similar results were obtained. Regarding locoregional recurrence (RR 0.79, 95% CI 0.22-2.78, *P* = 0.72) in patients, there was also no significant difference between with and without RAI ablation (Figure 3).

#### 3.3.2. Cancer Recurrence Rate in Patients with IR PTMC

We further performed data analysis and found that patients with intermediate-risk PTMC who with RAI ablation had a higher rate of cancer recurrence than those without RAI ablation (RR 0.23, 95% CI 0.11-0.49, *P* = 0.0001) (Figure 4). Furthermore, patients with risk factors for lymph node metastasis (RR 0.22, 95% CI 0.10-0.49, *P* = 0.0002), microscopic extrathyroidal extension (RR 0.21, 95% CI 0.07–0.65, *P* = 0.007), and multifocality (RR 0.15, 95% CI 0.04-0.53, *P* = 0.003) were more likely to have recurrence without RAI ablation (Figure 5). No significant statistical heterogeneity in treatment effects was observed in all meta-analyses, and all were statistically significantly different.

### 3.4. Analysis of Literature Publication Bias

An inverted funnel plot of the recurrence of RAI therapy in treating PTMC was produced to determine whether the articles had any publication bias. As Figure 6 shown, inverted funnel figure indicated publication bias in the research. The possible reasons were few literatures included in the meta-analysis and the heterogeneity between the articles. Subsequently, a subgroup analysis was performed that IR PTMC group have no publication bias.

## 4. Discussion

RAI ablation is an important adjuvant treatment for differentiated thyroid cancer after TT/NT [9]. However, two previous meta-analyses, both concluded that RAI ablation may not help reduce recurrence rates in PTMC patients [24, 25]. Unfortunately, there was heterogeneity in the results of both meta-analyses, and the researchers did not explore the source of the heterogeneity.

Our meta-analysis improved on the initial inclusion and exclusion criteria of the article. We excluded not only high-risk patients with macroscopic extrathyroidal extension, distant metastasis, or incomplete tumor resection but also studies with less than 5 years of follow-up. In addition, we only included studies in which the diagnostic criteria were structural recurrence. On the one hand, there is no accepted diagnostic criteria for biochemical recurrence. On the other hand, different studies had different definitions of cancer recurrence. Our uniform diagnostic criteria could reduce the impact on the meta-analysis results.

This meta-analysis of 8 retrospective studies including 2874 patients is evaluating whether RAI ablation reduces the likelihood of recurrence in patients with low- to intermediate-risk MPTC. The results showed that any recurrence rate with patients who had or had not received RAI ablation therapy was 2.87 versus 3.53%. The pooled analysis suggested that any cancer recurrence did not decrease with incremental RAI ablation. Pooled analysis showed that recurrence of any cancer did not decrease with increased RAI ablation. This finding was similar to the results of the two previous meta-analyses.

Unfortunately, the heterogeneity was found in the total meta-analysis (*P* = 0.0004, *I*^2^ = 76%), and we tried to investigate the reasons for the heterogeneity. We divided cancer recurrence into locoregional recurrence and distant metastasis, but the results were not as good as expected. Too few patients with distant metastasis could not be analyzed, while heterogeneity remained in the meta-analysis of locoregional recurrences. Therefore, we further divided the patients with LR-IR PTMC from the eight included studies into the IR PTMC group and the LR PTMC group. Since neither patient who underwent RAI ablation nor those who did not undergo RAI ablation in the two studies included in the LR PTMC group had cancer recurrence. So, we only analyzed whether RAI ablation in IR PTMC patients could reduce cancer recurrence. Fortunately, this subgroup lacked heterogeneity (*P* = 0.35, *I*^2^ = 8%) and was statistically different (*P* = 0.0001). In addition, we found that intermediate-risk patients with risk factors such as lymph node metastasis, microscopic extrathyroidal extension, and multifocality were more likely to recur in the absence of RAI ablation.

It is well known that microscopic extrathyroidal extension, lymph node metastasis, and/or multifocality are associated with increased recurrence rates [26–28]. Some scholars suggest that postsurgical PTMC should be treated with RAI like papillary thyroid carcinoma (PTC) larger than 1 cm [16, 18, 20, 21, 23]. While some other scholars are against it, arguing that it may be an overtreatment of PTMC patients [17, 19, 22]. It remains unclear whether RAI ablation in PTMC patients with these risk factors will reduce recurrence, which is now addressed by our meta-analysis.

There are several limitations to this meta-analysis. First, there are very few randomized clinical trials on the management of papillary thyroid cancer due to the inertness and longer survival rates of differentiated thyroid cancer and the associated high costs. Therefore, all included studies were retrospective. Second, our meta-analysis ensured that the recurrence of thyroid cancer is not influenced by the surgical approach and by high-risk factors, but many other factors influence its recurrence, such as the dose of iodine therapy and whether RAI ablation is complete. Third, the credibility of the results of our meta-analysis may be affected because of the small number of subgroups studied. Given the limitations of retrospective data meta-analysis in terms of methodology, a prolonged, randomized controlled trial with a greater sample size of patients could definitively address this issue.

## 5. Conclusion

According to the results of this meta-analysis, RAI ablation in IR PTMC patients who have already undergone surgery can significantly reduce thyroid cancer recurrence, especially when patients have some risk factors such as lymph node metastasis, microscopic extrathyroidal extension, and multifocality.

## Figures and Tables

**Figure 1:** Flowchart of study selection.

**Figure 2:** A forest plots that details any recurrence in LR-IR PTMC patients.

**Figure 3:** A forest plots that details the locoregional recurrence in LR-IR PTMC patients.

**Figure 4:** A forest plots that details the recurrence in patients with IR PTMC.

**Figure 5:** A forest plots that details the recurrence in PTMC patients with some risk factors (lymph node metastasis, microscopic extrathyroidal extension, and multifocality).

**Figure 6:** Funnel plot. SE: standard error; RR: risk radio.

**Table 1:** Cohort characteristics of included studies.

Study	Country	*N*	Mean age	Female/male	Mean tumor size (mm)	Histology	MF (%)	METE (%)	LNM (%)	Treat with RAI	RAI dose (mCi)	F/U year
Xue et al. [16]	China	137	NA	101/36	NA	PTMC	75.2	92.0	92.0	94	30-150	6.8
Kim and Kim [17]	Korea	704	47.0	631/73	6.0	PTMC	32.0	46.0	24.0	578	100	5.3
Creach et al. [18]	America	407	45.0	321/86	7.0	PTMC	46.2	NA	NA	NA	100	5.3
Neuhold et al. [19]	Austria	759	53.0	586/173	3.8	PTMC	31.2	NA	2.7	173	30	7.3
Moon et al. [20]	Korea	288	46.6	262/26	6.2	PTMC	20.5	30.9	33.7	114	30	6.0
Durante et al. [21]	Italy	312	47.5	277/35	5.0	PTMC	NA	0	0	137	73	6.7
Kim et al. [22]	Korea	307	46.0	275/32	8.0	PTMC	31.9	37.8	45.3	163	75-150	5.4
Chow et al. [23]	China	203	46.8	176/27	7.0	PTMC	31.0	20.7	24.6	137	80	8.4

PTMC: papillary thyroid microcarcinoma; LR: low risk; IR: intermediate risk; MF: multifocality; METE: microscope extrathyroidal extension; LNM: lymph node metastasis; RAI: radioiodine ablation, F/U: follow-up; NA: not available.

**Table 2:** Methodological quality assessment (risk of bias) of included studies by Newcastle–Ottawa scale.

References	Selection	Comparability	Outcome/exposure	Total score
Chow et al. [23]	★★★★	★✰	★★★	8
Kim et al. [22]	★★★★	★✰	★★★	8
Durante et al. [21]	★★★★	★★	★★★	9
Moon et al. [20]	★★★★	★✰	★★★	8
Neuhold et al. [19]	★★★★	★✰	★★★	8
Creach et al. [18]	★★★★	★★	★★★	9
Kim and Kim [17]	★★★★	★★	★★★	9
Xue et al. [16]	★★★★	★★	★✰★	8

A total of nine items were extracted, and each item was scored one “star.” The total scores ranged from 0 to 9.

## Data Availability

The data underlying the results presented in the study are available within the manuscript.
